The article "Effect of Applying Binocular Visual Training after Slanted Lateral Rectus Recession on Orthophoric Rate and Binocular Visual Function Recovery on Patients with Convergence Insufficiency-Type Intermittent Exotropia" was retracted in 2023. Reasons: unreliable results or conclusions; concerns about the data; concerns about the peer review; concerns about the citations.

# Effect of Applying Binocular Visual Training after Slanted Lateral Rectus Recession on Orthophoric Rate and Binocular Visual Function Recovery on Patients with Convergence Insufficiency-Type Intermittent Exotropia

**DOI:** 10.1155/2021/7202319

**Published:** 2021-10-16

**Authors:** Shuying Dai, Weifeng Sun, Hongjia Xu, Yanan Wang, Yuan Liu, Aijun Han, Lixiao Han, Juan Wang, Rujuan Liao, Sujiang Liu, Yu Gao, Huifang Han

**Affiliations:** Department of Strabismus and Pediatric Ophthalmology, Hebei Eye Hospital, Xingtai 054000, Hebei Province, China

## Abstract

**Objective:**

To explore the effect of applying binocular visual training after slanted lateral rectus recession on orthophoric rate and binocular visual function recovery on patients with convergence insufficiency-type intermittent exotropia (CI-IXT).

**Methods:**

A total of 76 CI-IXT child patients treated at the Strabismus and Pediatric Ophthalmology Department of our hospital from June 2019 to June 2020 were selected as the research objects, and those who met the inclusion criteria were equally divided into group A (63 eyes) and group B (61 eyes) according to the sealed envelope randomization. All child patients accepted the slanted lateral rectus recession, and after that, those in group A accepted the binocular visual training and those in group B accepted the conventional visual function rehabilitation training, so as to compare their position of eye, the best corrected visual acuity, etc., after training for statistical analysis.

**Results:**

Compared with group B after one month of surgery, group A had significantly less patients with grade I binocular vision function (*P* < 0.001) and more patients with grade II and III vision function (*P* < 0.05); between group A and group B, after 3 months and 6 months of treatment, the number of eyes with normal stereoscopic vision was significantly higher in group A (*P* < 0.05); at 15 days, 1 month, 3 months, and 6 months of treatment, the visual strain scores of group A were significantly lower (*P* < 0.001); after treatment, the number of orthophoria eyes was significantly higher in group A (*P* < 0.001), while the numbers of overcorrected eyes and undercorrected eyes were significantly higher in group B (*P* < 0.001); and the total incidence rate of adverse reactions was significantly lower in group A (*P* < 0.05).

**Conclusion:**

Applying binocular visual training to child patients with CI-IXT after slanted lateral rectus recession can promote the recovery of binocular vision and ensure higher safety, and further study will help to establish a better solution for the affected children.

## 1. Introduction

Intermittent exotropia (IXT) refers to the condition characterized by visual axis forming a divergent angle when looking at objects, which initially occurs when looking at objects in the distance, i.e., the patients are only able to intermittently control ocular alignment when looking at distant objects, whereas the visual axes of both eyes are often not in the same position [1, 2]. IXT affects as much as 1% of the population and often presents in childhood with rapid progression, of which the CI-IXT is a common type. Patients with CI-IXT can maintain orthophoria and stereoscopic vision in the early stage, but if effective and timely treatment is not adopted, constant exotropia may occurr once they cannot control the position of eye, seriously affecting their visual function [3] and causing serious visual dysfunction and psychological problems, especially in child patients. Therefore, effective correction of visual function is essential for stabilizing the position of the eye [4]. The slanted lateral rectus recession is a better way for correction of CI-IXT, but a more obvious lateral incomitance (LI) may occur after the surgery. Also, some scholars believe that [5] it may cause obvious postoperative drift in IXT patients, so it is suggested that postoperative visual correction measures shall be taken for patients accepting the slanted lateral rectus recession. Binocular vision training can promote the recovery of stereoscopic vision by correcting the anomalous retinal correspondence (ARC) and increasing the fusion function, with the effect that has been demonstrated in the reconstruction of postoperative binocular visual function in IXT children [6], but few studies have confirmed its efficacy in children with CI-IXT currently. Based on this, the effect of the aforesaid training on visual function in the affected children was explored in this study, with the results reported as follows.

The article "Effect of Applying Binocular Visual Training after Slanted Lateral Rectus Recession on Orthophoric Rate and Binocular Visual Function Recovery on Patients with Convergence Insufficiency-Type Intermittent Exotropia" was retracted in 2023. Reasons: unreliable results or conclusions; concerns about the data; concerns about the peer review; concerns about the citations.

## 2. Data and Methods

### 2.1. General Information

A total of 76 CI-IXT children treated at the Strabismus and Pediatric Ophthalmology Department of our hospital from June 2019 to June 2020 were selected as the research objects, and those who met the inclusion criteria were equally divided into group A (63 eyes) and group B (61 eyes) according to the sealed envelope randomization. The study was reviewed and approved by the Hospital Ethics Committee, and the statutory guardians of the affected children understood the purpose and process of the experimental study and signed the informed consent.

### 2.2. Inclusion and Exclusion Criteria

#### 2.2.1. Inclusion Criteria

① The patients met the diagnosis criteria for CI-IXT in the 7th edition of *The Wills Eye Manual* [7]; ② patients without cataracts, fundus diseases, amblyopia, glaucoma, fundus diseases, nystagmus, and other organic eye diseases; ③ the patients accepted the slanted lateral rectus recession; ④ according to the Burian typing [8], the exotropia of the patients was the convergence-insufficiency type (after 1 h of the diagnostic cover test, the exodeviation at near was over 15 PD); and ⑤ the patients were over 14 years of age.

#### 2.2.2. Exclusion Criteria

① Those who had poor comprehensive and understanding ability and who withdrew halfway; ② those who suffered from severe systemic diseases and could not go through the inspection and training; ③ those who presented with neurogenic disorders, growth retardation, and other diseases; ④ patients with a history of eye surgery and trauma, as well as a history of systemic diseases such as immune system and endocrine system diseases; and ⑤ patients with other types of strabismus, such as vertical strabismus, dissociative vertical strabismus, A-V pattern, paralytic strabismus, and restrictive strabismus.

### 2.3. Treatment Methods

The slanted lateral rectus recession was performed to children in both groups by the same surgical team. After surgery, children in group B accepted the conventional visual function rehabilitation training, a new pair of glasses was prescribed for each child by a professional optometrist for refraction correction, the routine quantitative cover was carried out, and by combining the family therapy with clinical treatment, an individualized diagnosis and treatment plan was made by the physician for the children to visit our clinic and finish corresponding tests and training. The specified fine training tasks including threading a needle, delineating practice, and stringing small beads were finished at home, the children revisited the clinic regularly, and their files were recorded [9, 10].

Children in group A accepted the binocular visual training after surgery with the Synoptophore MT-364 (manufactured: Shanghai Huanxi Medical Device Co., Ltd.) with the following methods. The first-grade training (simultaneous perception) was tested with the pictures of a lion and a cage; the second grade training (fusion) was tested with the pictures of cats and butterflies; and the third grade training (stereopsis) was tested with the pictures of San Mao, and the stereo image training was carried out. If the first-grade function was obtained, it was considered that the antisuppression treatment was finished; otherwise, visual flicker stimulation with the synoptophore should be repeated twice. Two weeks after surgery, the fusion pictures with cats and butterflies were used in the fusion training, which was performed by the way of combining, separating, moving in the lateral direction, and capturing. Each single training session lasted for 20 min, and the training was conducted once a day for continuous one week (one course) and then stopped for one week before the next course. The entire training lasted for continuous 6 months. Sensory and perceptual training: ① visual fixation stimulation: it referred to the exercise of looking at something for a period of time to project the seen object to the central fovea of retina, thereby improving the visual function; ② visual tracking: children were guided to look at an active object while keeping their head still to see if they could complete the tracking exercise successfully; ③ visual memory and reorganization: the visual memory and reorganization function of child patients were improved by playing fun games such as puzzle and magic cup game (figuring out which cup the object was under). The specified training plan should be made by combining with the vision recovery of child patients, and the contents should be properly adjusted according to their vision. Affected children in both groups received regular outpatient investigation and follow-up.

The article "Effect of Applying Binocular Visual Training after Slanted Lateral Rectus Recession on Orthophoric Rate and Binocular Visual Function Recovery on Patients with Convergence Insufficiency-Type Intermittent Exotropia" was retracted in 2023. Reasons: unreliable results or conclusions; concerns about the data; concerns about the peer review; concerns about the citations.

### 2.4. Observation Indexes

Examination of three grades of binocular vision function: the examination was conducted with the synoptophore; the first grade was tested with the pictures of lions and cages to record the simultaneous perception, self-conscious squint angle, and passive squint angle; the second grade was tested with the pictures of cats and butterflies to record the fusion function and range; and the third grade was tested with the pictures of San Mao to record the qualitative results of distance stereopsis. One month after surgery, the recovery of the child patients' binocular vision function was recorded.

The stereoscopic vision was inspected by the Titmus stereopsis test under natural light, the results of >80 arc-seconds were recorded as anomalous stereopsis, and the results of ≤60 arc-seconds were recorded as normal stereopsis.

The condition of visual strain of affected children at different moments was evaluated with the visual strain questionnaire [11], which covered the scoring items of reading, near work, headache, eye strain, and avoiding reading work (0 point indicating never, 1 point indicating sometimes, 2 points indicated often, and 3 points indicating always). The total score was 15 points, with higher scores denoting more serious visual strain.

Six months after treatment, the eye position of patients in both groups was evaluated as orthophoria (−8–0 PD), overcorrection (>0 PD) and undercorrection (>−8 PD), and their unaided visual acuity and the best corrected visual acuity after treatment were tested.

The article "Effect of Applying Binocular Visual Training after Slanted Lateral Rectus Recession on Orthophoric Rate and Binocular Visual Function Recovery on Patients with Convergence Insufficiency-Type Intermittent Exotropia" was retracted in 2023. Reasons: unreliable results or conclusions; concerns about the data; concerns about the peer review; concerns about the citations.

The incidence rates of adverse reactions of patients in both groups during follow-up were counted, including blood vessel congestion of palpebral conjunctiva, eye distension, headache, and orbital pain.

### 2.5. Statistical Methods

In this study, the professional data processing software was SPSS23.0, the picture drawing software was GraphPad Prism 7 (GraphPad Software, San Diego, USA), the enumeration data were examined with the *χ*^2^ test and expressed by [n (%)], the measurement data were examined by the *t*-test and expressed by mean ± SD, and differences were considered statistically significant at *P* < 0.05.

## 3. Results

### 3.1. Comparison of Baseline Information between the Two Groups

No significant differences in the gender ratio, mean age, preoperative strabismus angle, and other general information between the two groups were observed (*P* > 0.05), see Table 1.

### 3.2. Comparison of Recovery of Patients' Binocular Vision Function after One Month of Surgery between the Two Groups

Compared with group B after one month of surgery, group A had significantly less patients with grade I binocular vision function (*P* < 0.001) and more patients with grade II and III vision function (*P* < 0.05), see Table 2.

### 3.3. Comparison of Numbers of Eyes with Normal Stereopsis between the Two Groups at Different Moments

Before treatment, the numbers of eyes with normal stereopsis of groups A and B were 6 (9.52%) and 8 (13.11%), respectively. After 3 months of treatment, the numbers of eyes with normal stereopsis of groups A and B were 44 (69.84%) and 32 (52.46%), respectively. After 6 months of treatment, the numbers of eyes with normal stereopsis of groups A and B were 58 (92.06%) and 45 (73.77%), respectively. No significant difference in the numbers of eyes with normal stereopsis between the two groups before treatment was observed (*P* > 0.05), and after 3 months and 6 months of treatment, the numbers of eyes with normal stereopsis were significantly higher in group A than in group B (*P* < 0.05), see Figure 1.

### 3.4. Comparison of Visual Strain Scores between the Two Groups at Different Moments

At 15 days, 1 month, 3 months, and 6 months of treatment, the visual strain scores were significantly lower in group A than in group B (*P* < 0.001), see Table 3.

### 3.5. Comparison of Eye Position of Patients between the Two Groups after 6 Months of Treatment

Compared with group B after treatment, the number of orthophoria eyes was significantly higher (*P* < 0.001) and the numbers of overcorrected eyes and undercorrected eyes were significantly lower in group A (*P* < 0.05). See Table 4.

The article "Effect of Applying Binocular Visual Training after Slanted Lateral Rectus Recession on Orthophoric Rate and Binocular Visual Function Recovery on Patients with Convergence Insufficiency-Type Intermittent Exotropia" was retracted in 2023. Reasons: unreliable results or conclusions; concerns about the data; concerns about the peer review; concerns about the citations.

### 3.6. Comparison of Unaided Visual Acuity and the Best Corrected Visual Acuity between the Two Groups after Treatment

After treatment, the mean unaided visual acuity of groups A and B was (0.26 ± 0.01) and (0.44 ± 0.02), respectively. The mean best corrected visual acuity of groups A and B was (0.07 ± 0.01) and (0.17 ± 0.01), respectively. After treatment, the mean unaided visual acuity and the mean best corrected visual acuity were significantly lower in group A than in group B (*P* < 0.001), see Figure 2.

### 3.7. Comparison of Incidence of Adverse Reactions between the Two Groups during Follow-Up

The total incidence rate of adverse reactions was significantly lower in group A than in group B (*P* < 0.05), see Table 5.

## 4. Discussion

IXT is an ophthalmic disorder intermediate between phoria and strabismus, which often presents in childhood. Its pathogenesis is still unclear, but most scholars believe that fusion ability and decreased convergence function are the keys to its occurrence [12–14]. As a common type of IXT, CI-IXT not only affects the overall facial esthetics of child patients but also adversely affects the visual function of both eyes. In contrast to common strabismus, the fusion function and convergence function in CI-IXT children can be compensated, and their visual decompensation of both eyes is relatively late; hence, their visual function can be recovered more quickly after surgery [15, 16].

Clinical studies have confirmed that, after surgery, the convergence center function is still reduced in CI-IXT patients, and constant exotropia or even complete loss of stereopsis may occur in severe cases in case of no aggressive interventions [17, 18]. Currently, the slanted lateral rectus recession is a common surgical practice for treating CI-IXT, which modulates the visual axis of both the eyes to maintain balance and then restore the normal visual function of the affected children. However, it was documented [19] that surgical treatment alone had a higher rate of postoperative eye position regression, which would affect the recovery of visual function, and proper functional rehabilitation training after surgery will help patients to improve their convergence and fusion ability. In the past, synoptophore training was conducted to child patients for enhancing the fusion ability, correcting the retinal correspondence, and preventing eye position regression, which, although highly targeted, was time consuming and tedious; moreover, since most patients were children, the synoptophore training resulted in poor clinical compliance and ineffective interventions [20]. Recently, with the deeper exploration of human brain neuroplasticity, the medical community has introduced the concept of visual perception training into the rehabilitation training for amblyopia, strabismus, etc., and foreign scholars [21] have confirmed the efficacy of visual perception training in ameliorating the vision of strabismus patients. Research by YOON et al. [22] has also shown that, after IXT correction, early binocular vision training will help the recovery of stereoscopic function and binocular vision function by correcting the ARC and elevating the fusion ability. In this study, different visual training methods were adopted for the two groups of children after surgery, and the results showed that compared to group B, there were significantly fewer patients in group A with class I binocular visual function and significantly more patients with class II and III. This coincided with the abovementioned study and again confirmed the importance of binocular vision training for the reconstruction of binocular visual function in CI-IXT patients.

The article "Effect of Applying Binocular Visual Training after Slanted Lateral Rectus Recession on Orthophoric Rate and Binocular Visual Function Recovery on Patients with Convergence Insufficiency-Type Intermittent Exotropia" was retracted in 2023. Reasons: unreliable results or conclusions; concerns about the data; concerns about the peer review; concerns about the citations.

Binocular visual function, which is a higher-order visual function formed by humans in their perception of the external environment, refers to the process by which the visual cortex, when watching things with both eyes, identifies the physical image in the binocular macula retinae area and integrates the visual information from both eyes, thus forming the stereo image [23], whereas stereopsis, which is acquired by humans, is established on the basis of fusing vision and simultaneous perception. Stereopsis can help humans to gain a more comprehensive view of the three-dimensional space, which can be engaged in some relatively fine operations, and therefore, it is an important manifestation of binocular visual function [24, 25]. In this study, by combining with the previous experience of rehabilitation treatment, different vision training methods were adopted for the affected children of both groups after surgery, and according to the assessment of eye position and stereopsis condition of the research objects after 6 months of treatment, it was found that the orthophoria rate and the number of normal stereopsis cases were significantly higher in group A than in group B, which further proved that applying binocular visual training to CI-IXT children after the slanted lateral rectus recession could effectively improve the recovery of visual function and maintain postoperative orthophoria. By evaluating the binocular vision function in patients of both groups after one month of treatment, it was found that there were more patients with grade II and III vision function in group A than in group B, indicating that implementing binocular visual training to CI-IXT children after surgery could help them in reconstructing their visual function. But undeniably, the use of modern multimedia devices to carry out binocular vision training on children would have adverse effects; for instance, the electronic screen itself was injurious to the children's eyes. Also, the number of included cases was small, so this study was not fully representative and might lead to bias of the results, and the experimental design should be further refined in the future.

The article "Effect of Applying Binocular Visual Training after Slanted Lateral Rectus Recession on Orthophoric Rate and Binocular Visual Function Recovery on Patients with Convergence Insufficiency-Type Intermittent Exotropia" was retracted in 2023. Reasons: unreliable results or conclusions; concerns about the data; concerns about the peer review; concerns about the citations.

In conclusion, applying binocular visual training to CI-IXT children after the slanted lateral rectus recession can improve the orthophoria rate and promote the recovery of visual function. Further optimized training plans can benefit the affected children.

## Figures and Tables

**Figure 1:** Comparison of numbers of eyes with normal stereopsis between the two groups at different moments (eyes). *Note*. ^*∗*^Compared with group B, *P* < 0.05.

**Figure 2:** Comparison of unaided visual acuity and the best corrected visual acuity between the two groups after treatment (mean ± SD, LogMAR). *Note*. ^*∗*^The difference in the mean unaided visual acuity between the two groups after treatment was significant (*t* = 63.690, *P* < 0.001). #The difference in the mean best corrected visual acuity between the two groups after treatment was significant (*t* = 55.670, *P* < 0.001).

**Table 1:** Comparison of baseline information between the two groups.

Item	Group A (*n* = 38)	Group B (*n* = 38)	*χ* ^2^/*t*	*P*
Gender (n (%))			0.053	0.818
Male	21 (55.26%)	20 (52.63%)		
Female	17 (44.74%)	18 (47.37%)		

Mean age (mean ± SD, years)	8.31 ± 1.25	8.35 ± 1.32	0.136	0.893
Duration of disease (mean ± SD, years)	1.25 ± 0.36	1.28 ± 0.42	0.334	0.739
Preoperative strabismus angle (mean ± SD, ^△^)	−53.47 ± 6.84	−53.56 ± 6.78	0.058	0.954
Mean body weight (mean ± SD, kg)	27.21 ± 3.46	27.35 ± 3.52	0.175	0.862

Place of residence (n (%))			0.234	0.629
Urban area	14 (36.84%)	12 (31.58%)		
Rural area	24 (63.16%)	26 (68.42%)		

**Table 2:** Comparison of recovery of patients' binocular vision function after one month of surgery between the two groups (*n* (%)).

Group	*n*	I	III	III
Group A	38	4 (10.53)	13 (34.21)	21 (55.26)
Group B	38	21 (55.26)	5 (13.16)	12 (31.58)
*χ* ^2^		17.227	4.659	4.338
*P*		<0.001	<0.05	<0.05

**Table 3:** Comparison of visual strain scores between the two groups at different moments (mean ± SD, scores).

Group	*n*	Before treatment	15 days of treatment	1 month of treatment	3 months of treatment	6 months of treatment
Group A	38	11.26 ± 1.08	8.06 ± 1.23	7.28 ± 0.74	4.53 ± 0.51	3.17 ± 0.71
Group B	38	11.31 ± 1.14	9.72 ± 1.16	8.58 ± 0.62	6.26 ± 0.48	5.37 ± 0.67
*t*		0.196	6.052	8.301	15.227	13.892
*P*		0.845	<0.001	<0.001	<0.001	<0.001

The article "Effect of Applying Binocular Visual Training after Slanted Lateral Rectus Recession on Orthophoric Rate and Binocular Visual Function Recovery on Patients with Convergence Insufficiency-Type Intermittent Exotropia" was retracted in 2023. Reasons: unreliable results or conclusions; concerns about the data; concerns about the peer review; concerns about the citations.

**Table 4:** Comparison of eye position of patients between the two groups after 6 months of treatment (*n* (%)).

Group	Number of eyes	Orthophoria	Overcorrection	Undercorrection
Group A	63	54 (85.71)	7 (11.11)	2 (3.17)
Group B	61	33 (54.10)	19 (31.15)	9 (14.75)
*χ* ^2^		14.797	7.508	5.140
*P*		<0.001	<0.05	0.023

**Table 5:** Comparison of incidence of adverse reactions between the two groups during follow-up (*n* (%)).

Group	Number of eyes	Eye distension	Blood vessel congestion of palpebral conjunctiva	Headache	Orbital pain	Total incidence rate
Group A	63	2 (3.17)	0 (0.00)	1 (1.59)	1 (1.59)	4 (6.35)
Group B	61	3 (4.92)	2 (3.28)	4 (6.56)	2 (3.28)	11 (18.03)
*χ* ^2^						3.979
*P*						0.046

## Data Availability

The data used and analyzed during the current study are available from the corresponding author.

## References

[1] Mihara M., Hayashi A., Kakeue K. (2019). Longitudinal change in smooth pursuit in patients with intermittent exotropia after strabismus surgery. *Investigative Ophthalmology & Visual Science*.

[2] Ozates S., Ezerbolat Ozates M., Can C. U. (2019). Improvement in psychiatric symptoms after strabismus surgery in adolescent patients in long-term follow-up. *British Journal of Ophthalmology*.

[3] Bissen-Miyajima H., Ota Y., Nakamura K., Hirasawa M., Minami K. (2019). Binocular visual function with staged implantation of diffractive multifocal intraocular lenses with three add powers. *American Journal of Ophthalmology*.

[4] Nguyen J. H., Nguyen-Cuu J., Yu F. (2019). Assessment of vitreous structure and visual function after neodymium:yttrium-aluminum-garnet laser vitreolysis. *Ophthalmology*.

[5] Bennett C. R., Bex P. J., Merabet C. M. (2019). The assessment of visual function and functional vision. *Seminars in Pediatric Neurology*.

[6] Ma M. M., Kang Y., Chen C. (2021). Vision therapy for intermittent exotropia: a case series. *Journal of Optics*.

[7] Toro M. D., Reibaldi M., Longo A. (2019). Changes in visual function and ocular morphology in women who have undergone ART treatment and children born as a result of ART treatment: a systematic review. *Reproductive BioMedicine Online*.

[8] Ueda-Consolvo T., Ozaki H., Nakamura T., Oiwake T., Hayashi A. (2019). The association between cone density and visual function in the macula of patients with retinitis pigmentosa. *Graefes Archive for Clinical and Experimental Ophthalmology*.

[9] Tzameret A., Sher I., Edelstain V. (2019). Evaluation of visual function in Royal College of Surgeon rats using a depth perception visual cliff test. *Visual Neuroscience*.

[10] Andino D., Moy J., Gaynes B. I. (2019). Serum vitamin A, zinc and visual function in children with moderate to severe persistent asthma. *Journal of Asthma*.

The article "Effect of Applying Binocular Visual Training after Slanted Lateral Rectus Recession on Orthophoric Rate and Binocular Visual Function Recovery on Patients with Convergence Insufficiency-Type Intermittent Exotropia" was retracted in 2023. Reasons: unreliable results or conclusions; concerns about the data; concerns about the peer review; concerns about the citations.

[11] Tanimura N., Hatsusaka N., Miyashita H. (2019). Visual function and functional decline in patients with waterclefts. *Investigative Opthalmology & Visual Science*.

[12] Hiraoka M., Ohkawa E., Abe A. (2019). Visual function in mice lacking GM3 synthase. *Current Eye Research*.

[13] Jeon H., Jung J. H., Yoon J. A., Choi H. (2019). Strabismus is correlated with gross motor function in children with spastic cerebral palsy. *Current Eye Research*.

[14] Agarwal A. B., Cassinelli K., Johnson L. A. (2019). Seasonality of births in horizontal strabismus: comparison with birth seasonality in schizophrenia and other disease conditions. *Journal of Developmental Origins of Health and Disease*.

[15] Dotan G., Qureshi H. M., Toledano-Alhadef H., Azem N., Yahalom C. (2019). Prevalence of strabismus among children with neurofibromatosis type 1 disease with and without optic pathway glioma. *Journal of Pediatric Ophthalmology & Strabismus*.

[16] Cabrera M. T., Yanovitch T. L., Gandhi N. G., Ding L, Enyedi L. B (2019). The flipped-classroom approach to teaching horizontal strabismus in ophthalmology residency: a pilot study. *Journal of AAPOS: The Official Publication of the American Association for Pediatric Ophthalmology and Strabismus*.

[17] Raffa L. H., Fennell-Al Sayed H., LaRoche R. (2019). Measuring attention bias in observers of strabismus subjects. *Journal of AAPOS: The Official Publication of the American Association for Pediatric Ophthalmology and Strabismus*.

[18] Pineles S. L., Chang M. Y., Holmes J. M., Kekunnaya R., Özkan S. B., Velez F. G. (2019). Innovative techniques for the treatment of adult strabismus. *Journal of American Association for Pediatric Ophthalmology and Strabismus*.

[19] Europa T. A., Nel M., Heckmann J. M. (2019). A review of the histopathological findings in myasthenia gravis: clues to the pathogenesis of treatment-resistance in extraocular muscles. *Neuromuscular Disorders*.

[20] Baxter S. L., Nguyen B. J., Kinori M., Kikkawa D. O., Robbins S. L., Granet D. B. (2019). Identification and correction of restrictive strabismus after pterygium excision surgery. *American Journal of Ophthalmology*.

[21] Esaka Y., Kojima T., Dogru M. (2019). Prediction of best-corrected visual acuity with swept-source optical coherence tomography parameters in keratoconus. *Cornea*.

[22] Yoon L., Kim H.-Y., Kwak M. J. (2019). Utility of magnetic resonance imaging (MRI) in children with strabismus. *Journal of Child Neurology*.

[23] Gillies M. C., Hunyor A. P., Arnold J. J. (2019). Effect of ranibizumab and aflibercept on best-corrected visual acuity in treat-and-extend for neovascular age-related macular degeneration. *JAMA Ophthalmology*.

The article "Effect of Applying Binocular Visual Training after Slanted Lateral Rectus Recession on Orthophoric Rate and Binocular Visual Function Recovery on Patients with Convergence Insufficiency-Type Intermittent Exotropia" was retracted in 2023. Reasons: unreliable results or conclusions; concerns about the data; concerns about the peer review; concerns about the citations.

[24] Jabbarpoor Bonyadi M. H., Baghi A., Ramezani A., Yaseri M., Soheilian M. (2019). Correlation of macular thickness and visual acuity in DME treated by two doses of intravitreal ziv-aflibercept versus bevacizumab: analysis of a randomized, three-armed clinical trial. *Ophthalmic Surgery, Lasers and Imaging Retina*.

[25] Sousa K., Fernandes T., Gentil R., Mendonça L., Falcão M. (2019). Outer retinal layers as predictors of visual acuity in retinitis pigmentosa: a cross-sectional study. *Graefes Archive for Clinical and Experimental Ophthalmology*.

